The article "Metachronous tubulovillous and tubular adenomas of the anal canal" was published in 2015. Journal: Diagn Pathol.

# Metachronous tubulovillous and tubular adenomas of the anal canal

**DOI:** 10.1186/s13000-015-0379-9

**Published:** 2015-08-07

**Authors:** Hiroaki Nozawa, Soichiro Ishihara, Teppei Morikawa, Junichiro Tanaka, Koji Yasuda, Kensuke Ohtani, Takeshi Nishikawa, Toshiaki Tanaka, Tomomichi Kiyomatsu, Kazushige Kawai, Keisuke Hata, Shinsuke Kazama, Hironori Yamaguchi, Eiji Sunami, Joji Kitayama, Masashi Fukayama, Toshiaki Watanabe

**Affiliations:** Department of Surgical Oncology, The University of Tokyo, 7-3-1 Hongo, Bunkyo-ku, Tokyo 113-8655 Japan; Department of Pathology, The University of Tokyo, 7-3-1 Hongo, Bunkyo-ku, Tokyo 113-8655 Japan

## Abstract

Anal canal adenoma is an extremely rare disease that has the potential to transform into a malignant tumor. We herein presented a rare case of metachronous multiple adenomas of the anal canal. A 48-year-old woman underwent total colonoscopy following a positive fecal blood test. A 9-mm villous polyp arising from the posterior wall of the anal canal was removed by snare polypectomy. Histologically, the tumor was tubulovillous adenoma with high-grade dysplasia and the cut end was negative for tumor cells. Six years later, an elevated lesion, macroscopically five millimeters in size, was detected in the left wall of the anal canal in a follow-up colonoscopy. Local excision of the tumor was performed, and the lesion was pathologically confirmed to be tubular adenoma with high-grade dysplasia limited to the mucosa. The patient is currently alive without any evidence of recurrence for six months after surgery. Although she had a past history of cervical cancer, the multiple tumors arising in the anal canal were unlikely to be related to human papilloma virus infection. Our case report underscores the importance of careful observations throughout colonoscopy to detect precancerous lesions, particularly in anatomically narrow segments.

## Background

Anal canal tumors are a relatively uncommon occurrence in the context of all intestinal neoplasms. The predominant histology is the squamous cell type, whereas adenocarcinomas represent only 10 % of anal canal cancers [1–3], with adenomas in this segment being even more infrequent [1].

We herein described a patient with multiple anal canal adenomas that developed metachronously. Both lesions limited within the mucosa were removed in minimally invasive manners.

## Case presentation

A 40-year-old woman visited the Gynecological Department of our hospital with atypical genital bleeding for one and a half years. She was diagnosed with cervical cancer and subsequently underwent hysterectomy and bilateral salpingo-oophorectomy. Pathology of the resected cervix showed the non-keratinizing type of squamous cell carcinoma, measuring 2.5 × 2.5 cm in size, without nodal involvement (International Federation of Gynecology and Obstetrics (FIGO) Stage IB1). Immunohistochemistry revealed that the cancer cells were diffusely positive for p16 (CDKN2A) (Fig. 1).

**Fig. 1:** Immunohistochemical staining of p16 in cervical cancer (original magnification: 200 ×). Bar indicates 100 μm

During the follow-up, she was referred to our department at the age of 48 due to frequent anal bleeding after bowel movements. Laboratory blood tests showed no significant abnormalities; there were no signs of infection with hepatitis or human immunodeficiency viruses, and no elevations in the levels of the serum tumor markers carcinoembryonic antigen and carbohydrate antigen 19–9. A villous polyp was palpable on the posterior wall of the anal canal by a digital rectal examination. The polyp was just above the dentate line (Fig. 2a) and removed by snare polypectomy. The lesion was 9 × 5 mm in size and histologically diagnosed as tubulovillous adenoma with high-grade dysplasia, and the cut end was negative for tumor cells (Fig. 2b). Immunohistochemical staining revealed that almost all tumor cells were positive for Caudal-related Homeobox Transcription Factor 2 (CDX–2), whereas cytokeratin (CK)-7 staining was partially present. Moreover CK–20 immunoreactivity was only focally visible (data not shown).

**Fig. 2:** Findings of the first anal canal tumor. **a** Endoscopic appearance. **b** Histological appearance of a low magnification (original magnification: 20 ×). The border between adenoma and normal epithelium is indicated by a pair of arrowheads. Bar indicates 1 mm. The inset shows a higher-magnification view (original magnification: 200 ×)

The colon was regularly checked every year thereafter. At the age of 54, a follow-up colonoscopy showed another elevated lesion that developed from the left wall of the anal canal (Fig. 3a). The patient had anal discomfort after each bowel movement. She underwent transanal resection of the tumor. A pathological examination revealed tubular adenoma with high-grade dysplasia, approximately five millimeters in size (Fig. 3b). Immunohistochemical staining revealed that only a small number of tumor cells were positive for p16 (CDKN2A) (Fig. 3c). The patterns of CDX–2 and CK7/20 immunoreactivity were essentially the same as the first anal adenoma (data not shown).

**Fig. 3:** Findings of the second anal canal tumor. **a** Endoscopic appearance. **b** Histological appearance of a low magnification (original magnification: 40 ×). The border between adenoma and normal epithelium is indicated by an arrowhead. Bar indicates 1 mm. The inset shows a higher-magnification view (original magnification: 200 ×). **c** Immunohistochemical staining of p16 in the second anal canal tumor (original magnification: 200 ×). Only 4 % of tumor cells were positive for p16. Bar indicates 100 μm

The patient has remained free of recurrence seven months after tumor resection.

## Conclusions

Primary anal canal neoplasms are relatively rare. The most common histological type is squamous cell carcinoma that originates from the distal epithelium of this segment. On the other hand, adenocarcinomas only accounted for 10 % of anal canal malignancies [1–3]. They include two subtypes according to their origins: 1) mucosal-based adenocarcinomas that originate from colorectal-type epithelium at the proximal end of the anal canal, and 2) extra-mucosal adenocarcinomas arising from columnar epithelium lining of anal glands which open into the transitional zone. The latter is often associated with chronic fistulas [1–3]. Adenomas are distinctly rare entities in the anal canal; only a limited number of cases have been reported to date [4–7]. To the best of our knowledge, the present case is the first report in the literature on multiple anal canal adenomas. Based on the different directions of the tumor origins and the tumor-free margin of the first lesion, the two tumors are considered to have developed independently, and implantation of the first adenoma as a cause of the second tumor was unlikely. Furthermore, the CDX–2 positive phenotype indicates that both lesions of the anal canal were mucosal-based tumors, although the limited expressions of CK–7 and–20 were not typical profiles of colorectal adenomas [8].

Several recent case reports showed that definite adenocarcinomas arose from adenomas [6, 7]. These cases support the concept that the adenoma-carcinoma sequence, which is well recognized in colorectal carcinogenesis [9, 10], may be applicable to the development of adenocarcinoma in the anal canal.

Multiple etiological factors have been suggested to be associated with anal canal neoplasms such as anal intercourse, human immunodeficiency virus infection, and cigarette smoking [1, 11]. Furthermore, human papillomavirus (HPV) has been strongly implicated as a possible cause of tumorigenesis [12, 13]. Regarding histology, several studies showed that 78–92 % of squamous carcinomas and 40–43 % of adenocarcinomas were positive for HPV DNA [10, 14, 15]. Tachezy et al. reported that HPV positivity was also observed in 40 % of anal canal adenomas [14]. Our patient had a history of cervical cancer that was mostly linked to infection by HPV [16]. Taken together, we imagined that HPV infection might be a common cause of cervical cancer and metachronous anal canal tumors. Since the expression of p16 (CDKN2A), a cyclin-dependent kinase inhibitor, reliably reflects the status of HPV infection in various anogenital and head and neck malignancies [17, 18], we performed immunohistochemical staining of p16 in a resected specimen of the second anal canal tumor. However, immunoreactivity for p16 was negligible in the anal tumor cells, in contrast to the diffuse positivity observed in the cervical cancer cells. Our patient did not have other predisposing risk factors such as familial adenomatous polyposis, ulcerative colitis, or Crohn’s disease [4]. Therefore, we could not identify specific factors that may account for multiple tumorigenesis in the anal canal and cervix in our patient.

The prognosis of anal canal cancers remains unsatisfactory. The majority of these cancers are diagnosed in advanced stages that often require radical surgery such as abdominoperineal resection [2, 3]. Although multidisciplinary treatments have been introduced including surgery, chemotherapy, and radiation therapy, the five-year overall survival rate was estimated to be 39–63 % [2, 3, 19, 20]. Depth, lymph node metastases, histological grade, and radical surgery were previously identified as prognostic factors in anal canal cancers [2, 19, 21]. In our case, both lesions in the anal canal were pre-malignant and confined within the mucosa, suggesting a low risk of recurrence. Accordingly, the patient is now on follow-up without radiation or chemotherapy.

The present case underscores the importance of careful observations throughout colonoscopy to detect neoplastic lesions in the narrow segment that may potentially acquire an aggressive phenotype.

## Consent

Written informed consent was obtained from the patient prior to publication of this case report.

## Abbreviations

CDKN2A: Cyclin-Dependent Kinase Inhibitor 2A
CDX-2: Caudal-related Homeobox Transcription Factor 2
CK: Cytokeratin
FIGO: International Federation of Gynecology and Obstetrics
HPV: Human Papillomavirus
